# Analysis of the Effect of Quality Nursing on Recovery after Thoracic Surgery

**DOI:** 10.1155/2022/6204832

**Published:** 2022-10-07

**Authors:** Yujing Zhou, Ming Xu

**Affiliations:** Department of Thoracic Surgery, Shanghai Pulmonary Hospital Affiliated to Tongji University, Shanghai, China

## Abstract

**Objective:**

To observe the feasibility and safety of rapid rehabilitation nursing in the perioperative period of thoracoscopic treatment of lung cancer patients. Rapid rehabilitation nursing was compared with conventional perioperative nursing to explore its clinical efficacy, i.e., its advantages in improving postoperative comfort, postoperative rehabilitation efficiency, and hospitalization cost of patients undergoing thoracoscopic lung cancer resection.

**Methods:**

We carried out a retrospective analysis of 337 lung cancer patients who underwent lobectomy in our thoracic surgery department from July 2019 to June 2021, of which 168 lung cancer patients whose perioperative care method was traditional rehabilitation care were classified as *A* and 169 lung cancer patients who started to implement the intelligent medical intervention method in the department in September were classified as intelligent medical *B*. By reviewing patient cases and departmental statistics, general information, length of stay, hospitalization cost, complication rate, pain score, bowel movement recovery time, and pulmonary function index of the two groups *A* and *B* were compared. Nursing satisfaction was investigated by using a questionnaire. All the data in the study were processed and analyzed using SPSS 17.0 software.

**Results:**

There were no differences in preoperative general data, pathological findings, preoperative underlying diseases, lesion involvement sites, and postoperative TNM stages (*P* > 0.05), which were comparable; the incidence of postoperative pulmonary infection and atelectasis complications, postoperative hospitalization time, and hospitalization cost were lower in group *B* than in group *A*; the postoperative chest tube drain placement time was shorter in group *B* than in group *A*, and the difference between the two groups was statistically significant (*P* < 0.05). The incidence of postoperative pain and discomfort in group *B* was lower than that in group *A*, and the difference between the two groups was statistically significant (*P* < 0.05); the incidence of postoperative chest pain, bleeding, pneumothorax, pulmonary infection, and atelectasis in group *B* was lower than that in group *A*, and the difference between the two groups was statistically significant (*P* < 0.05).

**Conclusion:**

Intelligent medical rehabilitation nursing has good application value in thoracoscopic lung cancer surgery. Applying the concept of intelligent medical rehabilitation nursing provides an important experimental basis and theoretical basis for improving the postoperative survival quality and clinical symptoms of patients undergoing thoracoscopic lung cancer resection, which helps to promote the postoperative recovery of patients with thoracoscopic lung cancer, improves the recovery efficiency of patients and their overall quality of life, and is superior to the conventional nursing group.

## 1. Introduction

The incidence of lung cancer is increasing year by year due to the rapid development of society and the increasing and younger population of smokers. In western developed countries and industrialized cities in China, lung cancer accounts for the first place in malignant tumor incidence in men and the second or third place in women [1, 2], which has seriously threatened the health of all human beings. The histological types of lung cancer are generally divided into two categories: small cell carcinoma and non-small-cell carcinoma, of which non-small-cell lung cancer accounts for 80%, which also includes adenocarcinoma, squamous cell carcinoma, large cell carcinoma, and squamous adenocarcinoma [3, 4]. The clinical manifestations of lung cancer mainly include [5, 6] cough, bloody sputum, chest pain, fever, and symptoms of metastatic lung cancer foci. Most of the patients with intermediate- and late-stage cancer are exhibit severe cachexia and cancer pain in combination. Studies have shown that 35%–45% of patients with early and intermediate malignancy experience moderate or severe cancer pain, while 75% of patients in the progressive stage of the disease experience cancer pain of different degrees, of which 25%–30% suffer from severe cancer pain, especially for patients with advanced malignancy; nearly 80% of patients with intermediate and advanced lung cancer have obvious pain, so cancerous pain is a serious problem for tumor patients and medical workers [7, 8]. Cancer pain caused by lung cancer is one of the most important factors affecting the quality of life of lung cancer patients, most of who suffer from negative psychology, especially palliative care patients. Therefore, effective control of lung cancer pain is clinically important to improve patients' quality of life, which can make the last days of a patient's quality of life more dignified.

Lung cancer is one of the most common malignant tumor diseases in clinical thoracic surgery, and the most ideal treatment mode now is a comprehensive treatment mode based on surgery combined with radiotherapy and other treatment modalities [9, 10]. Among these, surgical treatment plays a leading role. At present, the main surgical methods for lung cancer are (1) wedge resection or partial resection; (2) lobectomy; (3) segmental resection; and (4) total pneumonectomy. The most common procedure performed at our hospital is lobectomy combined with lymph node dissection. Since the scope of surgical resection and trauma of lung cancer is much larger than that of ordinary pneumonectomy, lung function is often severely damaged and there are more postoperative complications. As surgery leads to loss of respiratory muscle, the proliferation of the elastic fiber layer of lung tissue, narrowing of the airway, and gradual reduction in the function of the airway mucosa result in a weakened endocrine elimination of the airway. Patients often develop respiratory dysfunction and other related complications after surgery. Patients are prone to postoperative complications such as bleeding, pneumothorax, pulmonary infection, and pulmonary atelectasis due to surgical trauma and anesthesia. Helping postoperative patients with lung cancer to effectively remove endocrine secretions from the airways is of positive significance to reducing the occurrence of postoperative complications and alleviating patients' postoperative pain, so effective perioperative nursing interventions are crucial to reduce the occurrence of postoperative complications in patients.

Intelligent medical is a concept that uses a series of optimized measures proven effective by evidence-based medicine in the perioperative period to accelerate patients' postoperative recovery. It focuses on the entire perioperative period, through a number of effective interventions for patients before, during, and after surgery, in order to shorten the patient's hospital stay, reduce hospital costs, reduce postoperative complications, and improve the efficiency of recovery. Perioperative care is an integral part of the intelligent medical concept and an important measure to improve patients' comfort. Studies have shown that active and effective intelligent medical rehabilitation care for lung cancer patients can effectively improve patients' respiratory function and reduce the incidence of postoperative complications in lung cancer patients [11], and nursing interventions play a key role in this treatment process [12]. However, the development of the nursing concept guided by the concept of intelligent medical rehabilitation surgery is relatively slow in its application in pulmonary surgery compared with other disciplines, and most clinical departments are still using traditional conventional nursing methods, which restricts the development and progress of intelligent medical rehabilitation surgery [13, 14]. In order to improve the understanding of the concept of intelligent medical rehabilitation nursing in the perioperative period of lung cancer, it is hoped that nursing staff can actively adopt this advanced nursing concept.

In this paper, we conducted a study on the application of intelligent medical rehabilitation nursing in the perioperative period of lung cancer patients and retrospectively analyzed 337 lung cancer patients who underwent lobectomy in our thoracic surgery department from July 2019 to June 2021, among which 168 perioperative lung cancer patients were treated with traditional rehabilitation and 169 lung cancer patients who started to adopt intelligent medical intervention methods in the department were classified as intelligent medical. The results found that intelligent medical rehabilitation care has good application value in thoracoscopic lung cancer surgery, and the application of the intelligent medical rehabilitation care concept provides an important experimental basis and theoretical basis for improving the postoperative survival quality and clinical symptoms of patients undergoing thoracoscopic lung cancer resection, which helps to promote the postoperative recovery of thoracoscopic lung cancer patients and improve the recovery efficiency of patients and their overall quality of life and is better than the conventional care group.

## 2. Materials and Methods

### 2.1. Sampling Method

A total of 337 lung cancer patients who underwent lobectomy at the Thoracic Surgery Department of Shanghai Pulmonary Hospital Affiliated with Tongji University from July 2019 to June 2021 were selected. 168 lung cancer patients who used traditional nursing methods in the perioperative period were selected as *A*, and 169 lung cancer patients who received intelligent medical nursing intervention methods after September 2020 were selected as intelligent medical as *B*.

### 2.2. Inclusion Criteria

1. According to the pathological staging criteria of lung cancer, all patients belonged to stage I–III patients with resectable lung cancer
2. None of them received radiotherapy or chemotherapy before surgery, and preoperative assessment could tolerate unilobe lobectomy
3. Preoperative CT examination showed that the patient had no hilar or mediastinal lymph node metastasis and no other malignant tumors
4. The patient has no functional lesions of important organs and no liver and kidney system diseases

### 2.3. Exclusion Criteria

1. Those with exploratory surgery or multilobectomy
2. Those with benign lung lesions
3. Those suffering from autoimmune diseases
4. Those who cannot cooperate with nursing intervention and observers due to cognitive impairment

### 2.4. Sample Size

Multivariate analysis in statistics generally requires that the sample size be 5 to 10 times that of the independent variable. This study expects up to 33 independent variables, so the required sample size is 165–330 cases. In this study, 300 cases were collected, and the sample size was increased by 10% to expand it to 337 cases.

### 2.5. Perioperative Management of Traditional Rehabilitation

According to the traditional nursing routine standards of thoracic surgery, perioperative management methods of traditional rehabilitation were as follows:

1. Admission education included medical history inquiry, ward environment introduction, safety knowledge (such as preventing falling from bed) related education, the introduction of a competent physician and nurse in charge, ward visiting time and visiting system introduction, diet-related knowledge education, and operation-related knowledge introduction.
2. Respiratory function exercise: the nurse in charge demonstrates and instructs the patient to perform respiratory function training, mainly with pursed lip abdominal breathing and balloon blowing. ① Pursed lip abdominal breathing: a combination of abdominal breathing and pursed lip breathing. The specific method is to assist the patient to take a sitting or semi-recumbent position, close the mouth and inhale deeply through the nose, then hold breath for 2–3 seconds, then slightly tilt chest forward, reduce the lips to a whistle-like shape, and breathe out through the mouth slowly, take a deep breath, and breathe out slowly. ② The blowing balloon method: the patient takes a deep breath, blows the balloon hard, stops for 1–2 seconds, and then removes the balloon.
3. Analgesic management: influenced by traditional concepts, patients do not use analgesics preventively after surgery. When the patient's NRS score is >4 points, 75–100 mg of laryngeal hydrochloride is administered intramuscularly for analgesia.
4. Early postoperative ambulation: according to traditional nursing routine, patients in the traditional rehabilitation lay flat on the first day after operation, take bedside X-rays, remove catheter on the second day, and assist in percussion on the back and expectoration, on the second day after operation. Three days later, according to the chest X-ray results, the chest drainage tube was removed and then patients could gradually get out of bed.

### 2.6. The Operation Method of Intelligent Medical Circle

Referring to “Guidelines for Intelligent Medical Surgery for Gastrectomy” by the European Association of Intelligent Medical Surgery, “Chinese Expert Consensus on Application of Intelligent Medical Surgery in Colorectal Surgery (2015 Edition)” by the Chinese Medical Association, and “China Intelligent Medical Surgery Periphery” issued by China Intelligent Medical Surgery Expert According to Expert Consensus on Operational Management (2016), combined with the characteristics of our department, we have made improvements in the following aspects of perioperative nursing interventions for lung cancer.

#### 2.6.1. On the Basis of Traditional Education for Patients in Intelligent Medical, Concept of Intelligent Medical Surgery and Pain Education Are Added

The specific method is as follows:

1. Outpatient consultation: during the outpatient consultation, the receiving physician will issue a publicity and education sheet for the introduction of perioperative knowledge. After entering the ward, a nurse in charge will introduce the basic content of the implementation of the concept of intelligent medical surgery and carry out publicity and education on lung cancer prevention. The hazards of smoking, inducing factors, pathogenesis, treatment methods, and prognosis of disease and key points of perioperative nursing and cooperation are explained to patients so that patients and their families have sufficient psychological preparation.
2. Missionary time: two focused missionary classes are held every Tuesday and Friday afternoon, and each class lasts two hours. Participants include patients and their families who are preparing for surgery. The lecturers are responsible nurses and head nurses, and the method is the slide show.
3. Propaganda and education content: in addition to the admission education content of *A*, perioperative knowledge of the concept of intelligent medical surgery will be introduced, and the advantages and importance of intelligent medical procedures will be explained through multimedia pictures and texts, so as to gain patients' understanding of intelligent medical care. The role of surgery and the current treatment level of hospitals and departments, pain-related knowledge, including pain score and pain medication, key points of cooperation before and after surgery, preoperative respiratory function training, and how to get out of bed early after surgery are explained, so that patients can get out of bed early. A good communication is established, and there is an exchange relationships with medical staff, and at the same time, through intensive publicity and education, they let patients get to know each other and understand each other, which is more conducive to patients to maintain a relaxed and comfortable psychological state. After propaganda class, responsible nurses with qualifications of psychological counselors in the department communicate inwards to find out the stressors of patients' nervousness and anxiety. By listing typical rehabilitation cases, patients are encouraged to enhance their confidence, eliminate doubts, actively cooperate with treatment, and focus on handover.

#### 2.6.2. Respiratory Function Training

The patients in intelligent medical were given a three-ball respiratory function trainer after admission and performed respiratory function training 4–6 times a day for 10 minutes each time. The main operation method is connecting the threaded connection tube of the lung function trainer to the interface and mouthpiece of the shell:

1. Inspiratory function training: first, place the base marked with the “Inhalation” mark, place it below, and place it vertically. Hold a mouthpiece and inhale deeply at a uniform and deep inspiratory flow rate to raise the float, while holding your breath for as long as possible, and then relax. Each inhalation training time is 10 to 15 minutes, and then return to normal breathing.
2. Exhalation function training: place the base marked with “Blowing” mark below, place it vertically, hold the mouthpiece, exhale evenly and deeply, raise the float, and do it for as long as possible. Hold, then relax, exhale for 10 to 15 minutes, and then resume normal breathing. After training, clean the trainer and put it away. At the same time, it is instructed to test tidal volume before the operation, record maximum inhalation and intake before the operation, and continue to use a respiratory function trainer to exercise respiratory function after operation. On the first day after operation, the patient began to practice using a respiratory function trainer, frequency was the same as that before operation, and the patient's physical strength was limited to the limit. The responsible nurse encouraged and supervised the patient to perform respiratory function training and assisted the patient to tap back and expel sputum.

In training of respiratory function, following points should be paid attention to the following:

1. All medical staff in the department should be proficient in using respiratory training devices. Before using it, they must explain to patients and their families that respiratory function training is very important to the success of the operation, strive for patients to understand the importance of respiratory function training for the operation and cooperate with medical staff to complete training. Medical staff should often go to ward off to encourage and urge patients to complete training, to ensure that each patient can use a respiratory function trainer proficiently and to ensure the time and frequency of daily exercise.
2. For preoperative patients with cardiovascular and cerebrovascular diseases, heart failure, and other diseases, it is necessary to observe the clinical manifestations of patients during respiratory function exercise. During the exercise of respiratory function, nurses gave corresponding guidance and supervision according to the specific situation of the patients and the training process was gradual to avoid adverse reactions such as respiratory muscle fatigue.

After one week of respiratory function exercise according to the above method, lung function was re-examined before the operation. It was found that values of MVV, FVC, and FEV1 were improved to different degrees after respiratory exercise and the difference was statistically significant (see Table 1 for specific values).

#### 2.6.3. Analgesic Management

The patients in intelligent medical were given preventive analgesics; that is, 5 mg of Tylenin was given orally TID on the first day after operation, and patients were observed for dizziness, constipation, nausea, and vomiting, and other reactions to other medicines.

Pain-related knowledge education is carried out before surgery, and pain assessment scales are posted in wards and corridors to teach patients to use pain scales correctly, including the following:

1. Definition of pain.
2. Causes of pain such as surgical injury and influence of disease itself.
3. Complications that may be caused by pain. For example, pain will affect postoperative coughing and deep breathing and may cause complications such as pneumonia and atelectasis.
4. Criteria and methods for pain assessment.
5. Common clinical analgesics, drug use methods and possible adverse reactions.
6. Teaching patients and their families to perform pain self-score. Postoperative chest pain was evaluated by pain numbers.

The NRS was used to fill in the pain nursing assessment sheet every day to evaluate the location, nature, and score of pain, the impact of pain on sleep, life, and mood, changes in the patient's treatment compliance, and whether there was constipation, nausea, and vomiting, skin itching, and other adverse reactions. Pain assessment sheets were written at 15 : 00 every day, identified by the patient's description of the most severe pain numerical score in the past 24 hours and linked to the previous day's pain score. The pain score is expressed in a digital form of 0–10 points, with 0 points indicating no pain, 1–3 points indicating mild pain (basically no pain when lying down quietly and not affecting sleep), 4–6 points indicating moderate pain severe pain (pain when lying down quietly, affecting sleep), and 7–9 points indicating severe pain (pain intolerable). Scores were continued 6 hours after surgery, on the 1st and 5th days after surgery, and the pain score scale was continued for 3 consecutive days after oral administration of Tylenine was stopped.

#### 2.6.4. Early Postoperative Ambulation

The patients in intelligent medical started to breathe deeply and coughed after waking up the day after operation. They changed their body positions in bed 6 hours after the operation. They started to sit by the bed in the morning on the first day after the operation, and then stood up (i.e., get out of bed trilogy).

Activity steps: assess the patient's general condition at the bedside, and if the condition is stable, assist in properly fixing the patient's chest closed drainage tube, subcutaneous negative pressure drainage tube, and other pipelines to avoid the drainage tube being folded, compressed, or prolapsed. Sit and lay down, encourage the patient verbally, assist him to slowly move his body to the bedside to sit and stand, first drop his legs for about 5 minutes, and observe whether the patient had symptoms such as dizziness, chest tightness, palpitations, sweating, and other symptoms, and the patient's response, if there is no discomfort, nurses and family members supported patient's bilateral armpits with both hands to assist him to stand up and stand firmly for 2-3 minutes. If there is no discomfort, assist the patient with bedside activities. After the patient gradually adapts, the patient can be supported to walk around the hospital bed for 3 to 5 minutes and gradually increase the amount of activity based on the general condition of the patient. It is not recommended to leave the ward during activities on the same day. If the patient can tolerate activity on the second day, it is recommended that family members and nurses are accompanied by the ward corridor andthe patient is prohibited from going downstairs. The amount of daily activity should be gradually increased according to the patient's physical strength. At the same time, strengthen the observation of the patient's condition to prevent falls.

### 2.7. Observation Indicators

The postoperative hospitalization days, hospitalization expenses, postoperative complication rate, bowel sound recovery time, postoperative pain numerical scale (NRS) score, and nursing satisfaction survey were observed. The changes in MVV, FVC, and FEV1 in intelligent medical at admission and the main indexes of pulmonary function were observed. The incidence of postoperative complications in patients was determined according to criteria for postoperative complications established by the US Centers for Disease Control and Prevention (CDC).

### 2.8. Data Collection Methods

General information, hospitalization time, hospitalization expenses, complication rate, pain score, bowel movement recovery time, and pulmonary function indexes were obtained by consulting the patient medical record system and department statistics. Questionnaire surveys and statistical analysis were performed.

## 3. Results

This study selected 337 lung cancer patients who underwent lobectomy in the Department of Thoracic Surgery, Shanghai Pulmonary Hospital, Tongji University, from July 2019 to June 2021. There were 168 lung cancer patients with traditional care methods during the perioperative period, including 100 adenocarcinomas and 68 squamous carcinomas, in 109 males and 59 females, aged 40–81 years, with a mean age of (57.22 ± 8.95) years. Smart medical (*B*) included 169 lung cancer patients who received a new rapid rehabilitation care intervention method after September 2019, including 113 adenocarcinomas and 56 squamous carcinomas, in 110 men and 59 women, aged 37–80 years, with a mean age (57.60 ± 10.23) years. There were no differences in general information such as gender, age, preoperative underlying disease, surgical site and method, postoperative pathology, and clinical TNM stage (*P* > 0.05), as shown in Table 2.

Patients in both conventional rehabilitation group *A* and smart medical group *B* successfully completed the corresponding single lobe resection and lymph node dissection. There were no cases of surgical death and no cases of secondary surgery within 30 days. The postoperative recovery time of bowel sounds was (26.12 V ± 3.34) hours for conventional rehabilitation *A* and (21.40 ± 2.60) hours for smart medical *B*. It was seen that the recovery time of bowel sounds shortened for smart medical patients. The postoperative hospitalization time was (11.98 ± 4.00) days for conventional rehabilitation *A* and smart medical *B*. The hospitalization cost of conventional rehabilitation A was (4.96 ± 1.22) thousand yuan and that of intelligent medical B was (4.36 ± 0.76) thousand yuan. The overall satisfaction score of nursing care for conventional rehabilitation *A* was (141.30 ± 2.62) points and that of intelligent medical *B* was (143.08 ± 2.03) points, which showed that the patient satisfaction improved with the adoption of intelligent medical care measures and the difference was statistically significant (*P* < 0.05) (Table 3).

The incidences of postoperative atelectasis and pulmonary infection in traditional rehabilitation *A* were 6.59% and 8.92%, respectively, while the incidences of postoperative atelectasis and pulmonary infection in intelligent medical *B* were 1.78% and 2.96%, which were lower. Compared with traditional rehabilitation, the incidence of arrhythmia in traditional rehabilitation *A* was 3.57% and the incidence of arrhythmia in intelligent medical *B* was 1.78%, which was lower than that in traditional rehabilitation, but there was no statistical significance (*P* > 0.05), as shown in Table 4.

The NRS scores of patients in traditional rehabilitation *A* were (6.02 ± 0.71) points and (5.88 ± 0.63) points 6 hours after operation and on the 1st day after operation, respectively. The NRS scores of patients in intelligent medical B were 6 hours after operation and on the first day after operation were (5.92 ± 0.70) and (5.72 ± 0.64) points, respectively. Due to the effect of the analgesic pump on the first day after operation, the NRS scores of patients in traditional rehabilitation *A* on the 2nd, 3rd, 4^th^, and 5th days after the operation were (4.92 ± 0.86), (3.81 ± 0.65), (3.29 ± 0.75), and (2.75 ± 0.67) points. The NRS scores of patients in intelligent medical *B* on the 2nd, 3rd, 4^th^, and 5th days after operation were (3.64 ± 0.78), (2.73 ± 0.72), (2.37 ± 0.59), and (1.87 ± 0.59) points, indicating that after scientific analgesia measures given after surgery, NRS scores of patients were lower than those of traditional rehabilitation, as shown in Table 5.

The patients in intelligent medical used a three-ball breathing trainer for respiratory function exercise after admission. The MVV, FVC, and FEV1 at admission were (111.13 ± 12.71) L/min, (3.51 ± 0.51) L, and (2.85 ± 0.39) L, respectively. The pulmonary function indexes MVV, FVC, and FEV1 of preoperative remeasurement were (131 ± 10.85) L/min, (3.66 ± 0.40) L, and (2.98 ± 0.33) L, respectively, which were improved compared with admission, indicating that the respiratory function trainer is of great significance to improve lung function of patients, as shown in Table 1.

## 4. Discussion

Lung cancer is the most common malignant tumor disease in clinical thoracic surgery, and thoracoscopic surgery is now the common means of treating lung cancer. Single port video-assisted thoracic surgery (SP-VATS) has the advantages of less surgical trauma, shorter hospital stay, and faster postoperative recovery, its surgical safety and 5-year survival rate are comparable to those of traditional thoracotomy, and it has been adopted by the National Comprehensive Cancer Network (NCCN) clinical treatment guidelines as a standard procedure for the treatment of early-stage lung cancer [15]. Because the extent of surgical resection and trauma for lung cancer is much greater than that of ordinary lobectomy, lung function is often severely impaired and postoperative complications are more frequent. Surgery leads to damage to respiratory muscles, proliferation of the elastic fibrous layer of lung tissue, narrowing of the airway, and progressive reduction in the function of the airway mucosa, resulting in reduced endocrine elimination of the airway, and respiratory dysfunction and other related complications usually occur in patients after surgery [16]. Some studies have demonstrated that giving lung cancer patients active and effective rapid rehabilitation nursing measures can effectively improve patients' respiratory function and reduce the incidence of postoperative complications in lung cancer patients. Active and effective rapid rehabilitation nursing interventions can effectively improve the respiratory function of lung cancer patients and have a positive effect on reducing complications and promoting recovery [17].

Currently, as an emerging concept, smart medicine has been applied in many surgical fields, especially in gastrointestinal surgery, with desirable results. The new nursing interventions guided by the theory of intelligent medicine mainly include a series of procedures, such as effective preoperative education and psychological care, new respiratory function training, effective analgesia, and early bed removal. The application of the smart medical concept in thoracic surgery lobectomy has proven to effectively reduce postoperative stress and shorten the hospital stay [18]. The hospitalization cost, postoperative pain score, and nursing satisfaction of patients guided by the smart medical concept were better than those of traditional rehabilitation, which is consistent with the results of the literature [19]. A study [20] found that active and effective preoperative mental health education can alleviate patients' anxiety and fears and enable them to receive surgical treatment in a good psychological state. A study [21] reported that the use of an intelligent medical rehabilitation surgical care model to intervene in the preoperative preparation of colon cancer patients could lead to voluntary medical care and reduce surgical complications. Clinical practice confirms that anxious and nervous psychological states may affect the effective implementation of the rapid rehabilitation model, that a good psychological state is an important factor in maintaining an individual's health, and that a patient's psychological state affects the speed of an individual's recovery. The model plays an important role [22]. Based on this theory, we have made the following improvements to the department's preoperative education and psychological intervention:

1. In terms of the time of education, traditional preoperative education starts with the patient's admission to the hospital, while the intelligent medical team's education time starts with the outpatient diagnosis so that patients and their families have a sufficient psychological preparation.
2. In terms of the content of education, the intelligent medical team began explaining the cause of the disease, treatment methods, the level of surgery in the department, the prognosis of the disease, and the current status and achievements of ERAS in the department in the form of slides and leaflets so that patients and their families can understand the disease. They have a correct understanding of the prognosis and gain support and cooperation.
3. In terms of psychological support, in addition to paying close attention to the psychological conditions of patients and their families, the smart medical team also identifies abnormal psychological conditions of patients in a timely manner and is guided by nurses in the department who are qualified as psychological counselors.

The incidence of postoperative pulmonary atelectasis and infection in smart medicine was 1.78% and 2.96%, respectively, which was lower than that of *T*-shaped radiation rehabilitation. Meanwhile, the comparison of various lung function indexes between patients' admission and preoperative lung function in smart medicine showed that patients' MVV, FVC, and FEV1 improved, suggesting that respiratory function trainers can improve patients' lung function and reduce postoperative lung function complications significantly. According to the basic principles of respiratory mechanics, there are fast breathing zones and slow breathing piers in human lung tissue. Due to postoperative pain and other reasons, patients have improper breathing patterns that allow gas to enter only the fast breathing zone of the lungs. After open heart surgery, the patient breathes less tidal volume, and at the same time, due to increased sputum secretion, fine bronchial constriction, or sputum not cleared in time, it is easy to cause complications such as pneumonia and pulmonary atelectasis. Therefore, effective respiratory function training in the perioperative period is important for the prevention of postoperative complications.

The NRS scores on postoperative days 2, 3, 4, and 5 were (3.64 ± 0.78), (2.73 ± 0.72), (2.37 ± 0.78). 0.59), and (1.87 ± 0.59) for the patients in smart medical *B*, respectively, which were lower than those of conventional rehabilitation, and the differences were statistically significant. This is consistent with the findings of [23] that postoperative multimodal analgesia can reduce postoperative pain scores. Open heart surgery is the most traumatic surgical procedure, and severe pain caused by surgical trauma and postoperative indwelling chest drains is the main cause of patients' stress reactions. Due to postoperative pain, patients have difficulty with sputum evacuation, restricted activities, depressed mood, and decreased immunity. Therefore, effective postoperative analgesia is especially important to accelerate patients' postoperative recovery. While the traditional concept of postoperative analgesia is to administer medication while the patient is in pain, the concept of smart medical surgery is multimodal analgesia and timed and scheduled medication. Due to the misunderstanding of traditional pain medication, some patients are reluctant to receive oral pain medication after surgery because they fear that taking pain medication will become addictive and affect postoperative wound healing. Pain education guided by the concept of smart medicine should focus on explaining to patients and families that short-term use of analgesics is not carcinogenic and is beneficial to postoperative recovery. Equipped with a portable pain scale, the content of pain education should be displayed with slides to ensure accurate and comprehensive understanding and acceptance by patients and their families.

The recovery time of postoperative bowel sounds in smart medicine was (21.40 ± 2.60) hours, which was shorter than the conventional rehabilitation, and the difference was statistically significant. One of the concepts of smart medicine is to get patients out of bed as early as possible after surgery, which can provide multiple psychological benefits to patients. A study [24] found that early postoperative bedtime activity improved splanchnic neuromodulation, promoted the recovery of gastrointestinal function, and prevented abdominal distension. A prospective randomized controlled study concluded that rapid postoperative rehabilitation of colorectal cancer patients to get out of bed and move around with exhaustion and defecation earlier than traditional rehabilitation methods promoted postoperative rehabilitation and recovery. However, in clinical work, medical staff and patients' families often consider the risk of postoperative complications, such as patients' weakness and early bed activity. Meanwhile, this study showed that the implementation of the trilogy did not increase the incidence of arrhythmias by getting out of bed, and the difference was not statistically significant. A study of 384 patients by foreign scholars found that early bed activity after gastrointestinal surgery did not increase the incidence of arrhythmias. There was a significant increase in the incidence of arrhythmias, falls, and other accidents. A study [25] of patients with resected bowel cancer also confirmed this idea. Getting out of bed as early as possible can accelerate blood circulation in the lower extremities, which can well prevent the occurrence of venous thrombosis in the lower extremities while maintaining the patient's good local skin and functional status. Early bed activity can also increase respiratory frequency, make secretions in the respiratory tract easier to discharge, reduce the occurrence of incisional infection, pulmonary atelectasis, and pleural effusion, promote lung recruitment, and improve patients' lung function.

In nursing interventions guided by the concept of smart medicine, emphasis is placed on helping patients get up early after surgery. Early waking up emphasizes that changing position as soon as possible on the day of surgery can effectively prevent the occurrence of upright hypotension, improve the patient's respiratory status, and promote the drainage of disease fluid if the patient's condition permits. From the first postoperative day, patients can sit and get up, thus promoting the recovery of peristalsis, reducing the occurrence of bloating and constipation, promoting blood return to the lower extremities, and reducing the risk of venous thrombosis of the lower extremities. With the increase in activity, the patient's bowel movement increases and the patient's appetite increases, which helps improve the nutritional status of the deceased, facilitate tissue repair and incision healing, enhance the patient's own self-care ability, and make the patient recover better after surgery. Optimistic awareness can accelerate the recovery process of patients, minimize the number of escorts, and reduce the burden and pressure on patients' families and is also important for shortening the number of treatment days and reducing hospitalization costs.

## 5. Conclusion

First, intelligent medical rehabilitation nursing has good application value in the postoperative recovery of thoracoscopic lung cancer surgery patients, and the application of its concept is safe and feasible.

Second, the intelligent medical rehabilitation nursing model in the postoperative recovery of patients undergoing thoracoscopic lung cancer surgery reduces patients' pain, decreases the incidence of postoperative complications, shortens the retention time of chest drains, improves patients' comfort during the perioperative period, and reduces the number of hospital days and hospitalization costs, and this nursing intervention is better than conventional nursing.

Third, the implementation of the intelligent medical rehabilitation care model can help promote the postoperative recovery of patients undergoing thoracoscopic lung cancer surgery and improve the overall quality of life of patients.

## 6. Prospects and Shortcomings

First, in the context of the current postoperative management of lung cancer, the development of the intelligent medical rehabilitation nursing model improves the efficiency of patient recovery, gives patients more effective measures for perioperative nursing interventions, helps improve their survival quality, and provides an important experimental basis and theoretical basis for improving the postoperative survival quality or clinical symptoms of patients undergoing thoracoscopic lung cancer resection, which is worthy of further clinical application and promotion.

Secondly, the shortcomings of this study are that the research method is retrospective, with large bias, rough, and often inaccurate due to incomplete records, increased errors, subjective factors, and other shortcomings such as the inability to compare the observation group with the control group simultaneously and perform random sampling for the sample source. So the next study should also screen and include more cases that meet the criteria for more in-depth analysis and fully incorporate consideration of postradiotherapy treatment to draw more meaningful conclusions and provide an important reference for intelligent medical rehabilitation care treatment of lung cancer.

## Figures and Tables

**Table 1:** Comparison of pulmonary function indexes of patients in accelerated rehabilitation before admission and operation.

Project	Company	Admission (*n* = 169)	Preoperative (*n* = 169)	*P* value
MVV (maximum minute ventilation)	L/min	111.15 ± 12.72	131.02 ± 10.87	<0.001
FVC (forced vital capacity)	L	3.52 ± 0.53	3.68 ± 0.42	0.003
FEV1 (forced expiratory volume in first second)	L	2.86 ± 0.37	2.96 ± 0.35	0.001

**Table 2:** Comparison of general data of patients.

Project	Content	*A* (*n* = 168)	*B* (*n* = 169)	*P*
Age	Year	57.23 ± 8.96	51.61 ± 10.24	0.718

Gender	Male	109 (64.8%)	110 (65.3%)	0.969
	Female	59 (35.2%)	59 (34.8%)	—

Pathology	Adenocarcinoma	100 (59.6%)	113 (66.7%)	0.164
	Squamous cell carcinoma	68 (41.4%)	56 (33.3%)	

Basic diseases	Hypertension	34 (20.5%)	28 (18.5%)	0.836
	Coronary heart disease	16 (9.3%)	21 (13.5%)	
	Diabetes	21 (12.3%)	18 (11.4%)	

Lesion location	Upper lobe of the right lung	45 (26.5%)	61 (36.3%)	0.055
	Middle lobe of the right lung	12 (7.3%)	11 (6.6%)	
	Right inferior lobe of the lung	45 (26.5%)	34 (20.2%)	
	Upper lobe of the left lung	32 (19.1%)	43 (25.5%)	
	Left inferior lobe of the lung	34 (20.3%)	20 (11.9%)	

Pathological stage	IA	36 (21.2%)	34 (20.3%)	0.882
	IB	43 (25.3%)	39 (23.3%)	
	IIA	30 (17.6%)	37 (21.7%)	
	IIB	32 (19.3%)	30 (17.8%)	
	IIIA	27 (16.3%)	29 (17.3%)	

**Table 3:** Comparison of bowel sounds recovery time, postoperative hospitalization time, hospitalization expenses, and nursing satisfaction.

Project	Company	*A* (*n* = 168)	*B* (*n* = 169)	*P* value
Bowel sound recovery time	Hours/h	26.15 ± 3.31	21.41 ± 2.61	<0.001
Postoperative hospital stay	Days/d	11.99 ± 4.01	8.92 ± 2.44	<0.001
Hospitalization expenses	Ten thousand	4.95 ± 1.24	4.34 ± 0.77	<0.001
Nursing satisfaction	Minute	141.33 ± 2.61	143.05 ± 2.05	<0.001
Comprehensive score				

**Table 4:** Comparison of postoperative complications.

Postoperative complications	*A* (*n* = 168)		*B* (*n* = 169)		*P* value
	Number of cases	Incidence rate (%)	Number of cases	Incidence rate (%)	
Atelectasis	10	6.58	4	1.77	0.031
Pulmonary infection	15	8.93	5	2.95	0.021
Arrhythmia	7	3.55	3	1.79	0.247
Total	32	19.05	10	6.50	0.009

**Table 5:** Comparison of postoperative pain scores.

Category	*A* (*n* = 168)	*B* (*n* = 169)	*P* value
6 hours after surgery	6.03 ± 0.72	5.94 ± 0.72	0.215
Day 1 after surgery	5.87 ± 0.61	5.71 ± 0.65	0.026
Day 2 after surgery	4.94 ± 0.85	3.65 ± 0.77	<0.001
Day 3 after surgery	3.82 ± 0.66	2.71 ± 0.74	<0.001
Day 4 after surgery	3.27 ± 0.77	2.35 ± 0.61	<0.001
Day 5 after surgery	2.77 ± 0.66	1.89 ± 0.57	<0.001

## Data Availability

The simulation experiment data used to support the findings of this study are available from the corresponding author upon request.
